# DNA methylation-mediated repression of exosomal miR-652-5p expression promotes oesophageal squamous cell carcinoma aggressiveness by targeting PARG and VEGF pathways

This article has been retracted.

**DOI:** 10.1371/journal.pgen.1008592

**Published:** 2020-04-28

**Authors:** Peng Gao, Dan Wang, Meiyue Liu, Siyuan Chen, Zhao Yang, Jie Zhang, Huan Wang, Yi Niu, Wei Wang, Jilong Yang, Guogui Sun

**Affiliations:** 1 Department of Bone and Soft Tissue Tumor, Tianjin Medical University Cancer Institute and Hospital, National Clinical Research Center for Cancer, Key Laboratory of Cancer Prevention and Therapy, Tianjin's Clinical Research Center for Cancer, Tianjin Medical University Cancer Institute and Hospital, Tianjin, China; 2 Department of Radiation Oncology, North China University of Science and Technology Affiliated People's Hospital, Tangshan, China; 3 Department of Pathology, North China University of Science and Technology Affiliated People's Hospital, Tangshan, China; Novartis, UNITED STATES

## Abstract

Exosomal microRNAs (miRNAs) have been recently shown to play vital regulatory and communication roles in cancers. In this study, we showed that the expression levels of miR-652-5p in tumour tissues and serum samples of oesophageal squamous cell carcinoma (OSCC) patients were lower compared to non-tumorous tissues and serum samples from healthy subjects, respectively. Decreased expression of miR-652-5p was correlated with TNM stages, lymph node metastasis, and short overall survival (OS). More frequent CpG sites hypermethylation in the upstream of miR-652-5p was found in OSCC tissues compared to adjacent normal tissues. Subsequently, miR-652-5p downregulation promoted the proliferation and metastasis of OSCC, and regulated cell cycle both in cells and *in vivo*. The dual-luciferase reporter assay confirmed that poly (ADP-ribose) glycohydrolase (PARG) and vascular endothelial growth factor A (VEGFA) were the direct targets of miR-652-5p. Moreover, the delivery of miR-652-5p agomir suppressed tumour growth and metastasis, and inhibited the protein expressions of PARG and VEGFA in nude mice. Taken together, our findings provide novel insight into the molecular mechanism underlying OSCC pathogenesis.

## Author summary

This study confirmed that miR-652-5p underexpression was a result of the hypermethylated promotor, which regulated OSCC development by targeting PARG and VEGF. Serum miR-652-5p might be used as a potential tumour marker to predict the OS of OSCC patients. The miR-652-5p gene may be a suppressor gene in OSCC, which serves as a potential therapeutic target for OSCC.

## Introduction

Oesophageal cancer is a commonly diagnosed malignancy in the digestive system with high incidence and mortality. WHO statistics showed that it ranks as the 4th highest cause of cancer death worldwide with 400,000 deaths and 456,000 new cases in 2012, and over 50% of the new cases were found in China [1,2]. Recent development in diagnostic and treatment strategies, such as the combination of surgery, radiation and/or chemotherapy, have improved the prognosis of patients with oesophageal squamous cell carcinoma (OSCC) [3–5]. However, due to the absence of specific and sensitive biomarkers, and the lack of typical signs and symptoms, OSCC is often diagnosed at late stages, and the 5-year survival rate is lower than 15%. Thus, investigations on the molecular mechanisms involved in OSCC progression and the development of novel therapeutic strategies for OSCC patients are urgently needed.

MicroRNAs (miRNAs) are a group of small noncoding RNAs (18–25 nucleotides) that bind to target mRNAs, resulting in either degradation or translation inhibition, and eventually silencing of these mRNAs [6,7]. The dysfunction of miRNAs has been reported in various types of cancers including OSCC. Emerging evidence has also shown that miRNAs exist both in cells and circulating blood, which may reflect the conditions of tissues or organs. Circulatory miRNAs remain stable in blood because of their resistance to the degradation by RNase enzymes [8], suggesting that they may serve as potential diagnostic or prognostic biomarkers. The potential use of miRNA in the early detection of different human malignancies has been previously reported, such as pulmonary cancer [9], breast cancer[10] and stomach cancer [11]. The main reason why circulatory miRNAs remain undegraded is that these miRNAs are encapsulated in extracellular membrane vesicles, such as exosomes [12], which are small vesicles (30–150 nm) that have been recognized as a key player in intercellular communication [13,14]. Recent data showed that exosomes played essential roles in regulating tumour-microenvironment crosstalk via the horizontal transfer of mRNAs, miRNAs, and proteins [15,16]. Tumour-specific exosomes are secreted from tumour cells and then enter circulation, indicated that exosomal miRNAs in body fluids may become useful diagnostic markers in cancer detection [17]. However, little is known about the relationship between circulatory exosomal miRNA and the pathogenesis of OSCC.

MiR-652-3p and miR-652-5p are two highly conserved miRNAs belonging to the mammalian miR-652 family, which is located in chromosome Xq23. Recent findings revealed that miR-652-5p might be a promising prognostic biomarker in patients with locally advanced oesophageal adenocarcinoma [18]. However, the regulatory impact of miR-652-5p in OSCC remains to be elucidated. In the current study, we assessed the expression level of miR-652-5p and its prognostic significance in OSCC. The correlation between miR-652-5p level and OSCC development, and the role of serum miR-652-5p as a non-invasive biomarker in OSCC were explored. The mechanism underlying the regulation of miR-652-5p in tumour growth and metastasis was also investigated.

## Results

### Decreased miR-652-5p expression is associated with poor survival in OSCC patients

To identify the potential function of miR-652-5p in OSCC, the expression level of miR-652-5p in OSCC tissue samples (n = 93) and paired adjacent normal tissues(n = 93) were analysed. OSCC tissues showed negative or weak miR-652-5p staining, whereas normal tissues presented light to dark colour (Fig 1, Table 1). The miR-652-5p signal was confined to scattered in the positive images of tumour tissues (Fig 1A and 1B). The expression of miR-652-5p was significantly decreased in tumour tissue samples, especially the ones from OSCC stages III and IV, as compared to the controls (Fig 1C and 1D). The downregulation of miR-652-5p was associated with OSCC stages and lymph node metastasis (Table 1). Also, the overall survival (OS) of patients was significantly shorter in the ones with low miR-652-5p expression (Fig 2A).

**Fig 1:** Detection of miR-652-5p expression in OSCC and adjacent normal tissues. **(A)**Scrambled miRNA and **(B)** U6 snRNA as negative and positive controls, respectively. Expressions of miR-652-5p in **(C)** adjacent normal tissues (n = 93) and **(D)** OSCC samples (n = 93; middle: moderate or low expression, left and right: no or low expression).

**Fig 2:** MiR-652-5p level in OSCC tissues and serum samples. **(A)**Kaplan–Meier OS curves of low and high expressions of miR-652-5p in OSCC patients (n = 93). **(B)** Quantitative analysis of miR-652-5p expression level in paired OSCC samples (n = 100) and corresponding normal tissues (n = 100). **(C-D)** The expression of miR-652-5p in lymph node metastasis and different stages of OSCC. **(E)** Kaplan-Meier curve shows the OS of OSCC patients according to miR-652-5p expression. (**F)** The expression level of miR-652-5p in the serum samples of OSCC patients (n = 110) and healthy subjects (n = 57). **(G-H)**The expression of miR-652-5p in patients with lymph node metastasis and at different stages. **(I)** ROC curve analysis of miR-652-5p level for the detection of OSCC.

**Table 1:** Correlation between miR-652-5p expression and clinicopathological parameters of OSCC patients.

Characteristics	Training group (n = 93)			Test group (n = 100)		
	Low (n = 72)	High (n = 21)	*P*	Low (n = 74)	High (n = 26)	*P*
Gender						
Male	59 (76.6%)	15 (23.4%)	0.293	62 (74.7%)	21 (25.3%)	0.316
Female	13 (68.4%)	6 (28.6%)		10 (66.7%)	5 (23.3%)	
Age						
≤60	22 (81.5%)	5 (18.5%)	0.549	25 (73.5%)	9 (26.5%)	0.939
> 60	50 (75.8%)	16 (24.2%)		49 (74.2%)	17 (25.8%)	
Tumor size						
< 5 cm	41 (80.4%)	10 (19.6%)	0.450	50 (76.9%)	15 (23.1%)	0.364
≥ 5 cm	31 (73.8%)	11 (26.2%)		24 (68.6%)	11 (31.4%)	
Tumor stages^a^						
T1+ T2	16 (72.2%)	6 (27.3%)	0.605	14 (60.9%)	9 (39.1%)	0.102
T3+ T4	50 (78.1%)	14 (21.9%)		60 (77.9%)	17 (22.1%)	
Histological grade						
Well/moderate	57 (77.0%)	17 (23.0%)	0.858	62 (75.6%)	20 (24.4%)	0.433
Poor/NS	15 (78.9%)	4 (21.1%)		12 (66.7%)	6 (33.3%)	
Lymph node metastasis						
Negative	27 (60.0%)	18 (40.0%)	0.000	39 (66.1%)	20 (33.9%)	0.031
Positive	45 (93.8%)	3 (6.2%)		35 (85.4%)	6 (14.6%)	
Clinical stages^a^						
I + II	30 (62.5%)	18 (37.5%)	0.000	36 (62.1%)	22 (37.9%)	0.000
III + IV	38 (77.3%)	2 (22.7%)		38 (90.5%)	4 (9.5%)	

^a^Numbers might be less than the total number if missing data.

The mRNA level of miR-652-5p in OSCC tissues, particularly the ones from patients at advanced stages or with lymph node metastasis, was remarkably lower than that in normal samples (Fig 2B), (Fig 2C and 2D, Table 1). The underexpression of miR-652-5p was associated with the poor prognosis of OSCC patients (Fig 2E). Data also showed that miR-652-5p was an independent prognostic factor for the OS of OSCC patients (S1 Table).

The serum expression of miR-652-5p in OSCC patients was significantly lower in comparison to the controls (Fig 2F, S2 Table). The serum level of miR-652-5p was negatively correlated with the lymph node metastasis and advanced stages of OSCC (Fig 2G and 2H, S2 Table). The receiver operating characteristic (ROC) curve showed that the area under the curve (AUC) for plasma miR-652-5p was 0.919, indicating the diagnosis potential of serum miR-652-5p for OSCC (Fig 2I).

Exosomes were collected from the serum of all participants. They appeared with a round shape morphology with 100 nm in size, and showed positive staining for the two exosomal markers, CD63 and CD81(Fig 3A–3D). The expression of exosomal miR-652-5p in OSCC patients was reduced as compared to healthy participants (Fig 3E).

**Fig 3:** Analyses of serum exosomes and exosomal miRNAs. **(A-B)** The detection of surface markers CD63 and CD81 in serum exosomes from OSCC patients and healthy participants.**(C-D)** Size detection of serum exosomes. **(E)** miR-652-5p level in serum exosomes was measured by qRT-PCR. Results from triplicate experiments are shown.Data are presented as the mean ± SD from triplicate experiments.

### DNA hypermethylation leads to miR-652-5p downexpression in OSCC

Next, we detected CpG sites methylation using the MassARRAY System. MiR-652-5p promoter contained CpG sites, suggesting that DNA methylation might be involved in the modulation of miR-652-5p transcription. The amplicon (558 base pairs long) in the promoter region of miR-652-5p consisted of 20 CpG sites that could be divided into 13 units. The level of CpG methylation was detected based on the colour of each miR-652-5p CpG unit in individual sample. Data showed that the methylation status of miR-652-5p in tumorous tissues was different from that in normal samples (Fig 4A). By using hierarchical clustering analysis, we observed that the density of methylated CpG dinucleotides was increased in OSCC samples compared to paired normal tissues (Fig 4B). Also, the methylation levels of 13 CpG units (except for CpG7 and CpG9) within the miR-652-5p promoter were much higher in OSCC tissues versus normal samples (Fig 4C). OSCC tissues also showed significantly higher methylation levels of CpG1, CpG2.3.4, CpG5, CpG6, CpG8, CpG10, CpG11, CpG12, CpG13.14, CpG15, CpG16.17, CpG18.19, and CpG20 (mean methylation = 41.10%, 43.44%, 23.94%, 32.83%, 44.39%, 47.06%, 21.89%, 36.61%, 43.67%, 35.00%, 41.50%, 43.06%, and 37.39%, respectively) compared to normal tissues samples (mean methylation = 21.72%, 18.89%, 7.17%, 16.94%, 15.67%, 11.56%, 10.83%, 13.72%, 18.17%, 11.67%, 22.50%, 17.06%, and 17.78%, respectively).

**Fig 4:** Methylation of miR-652-5p. **(A)**The methylation profile of CpG sites in miR-652-5p. The percentage of methylation in each site was indicated by different colours. Boxes show different methylation patterns in OSCC (n = 18) and corresponding normal tissue samples (n = 18). **(B)** Hierarchical cluster analysis shows CpG sites methylation in miR-652-5p promoter region in 18 OSCC and normal tissue samples. The colour gradient indicates the methylation level (0% to 100%) of each unit in each sample. **(C)** The distribution of thirteen analysed CpG units in miR-652-5p promoter. **(D)** Methylation level of miR-652-5p promoter in OSCC cells treated with 5-Aza-CdR. **(E)** Quantitative measurement of miR-652-5p level in 5-Aza-CdR-treated cells. Data from triplicate experiments are presented.

Later, cells were treated with the demethylation agent 5-aza-2-deoxycytidine (5-aza-CdR). The methylation of miR-652-5p in EC109 (41.94% vs. 17.70%) and KYSE150 (51.19% vs. 23.02%) cells were predominantly inactivated at the presence of 5-aza-CdR (Fig 4D). Correspondingly, the high expression of miR-652-5p was negatively correlated with the methylation level in these 5-aza-CdR-treated cells (Fig 4E). These findings implied that miR-652-5p downregulation in OSCC was correlated with promoter hypermethylation, while the demethylation of the promoter gene induced the upregulation of miR-652-5p.

### miR-652-5p suppresses OSCC cell growth and metastasis

Among the tested OSCC cells, EC109 and KYSE150 showed the lowest miR-652-5p expression (Fig 5A) and were used for the overexpression study. EC109 and KYSE150 cells were transfected with miR-652-5p mimic followed by the measurement of miR-652-5p level using qRT-PCR. The transfection efficiency was verified using qRT-PCR, which showed a remarkable elevation of miR-652-5p expression in EC109 and KYSE150 cells (Fig 5B). Upregulated exogenous expression of miR-652-5p efficiently impeded the growth, colony formation, and migration/invasion of OSCC cells (Fig 5C–5H). Next, flow cytometry was performed to better understand the inhibitory role of miR-652-5p in cell growth. Data showed an increased number of cells in G0/G1 phase upon upregulation of miR-652-5p in both EC109 and KYSE150 cell lines (Fig 5I and 5J), suggesting that miR-652-5p overexpression led to G1 phase arrest in OSCC cells.

**Fig 5:** miR-652-5p overexpression suppressed cell proliferation, colony formation and migration. (A) The level of miR-652-5p in OSCC cells. (B) The miR-652-5p level in miR-652-5p mimic-transfected EC109 and KYSE150 cells. (C-D) The growth of miR-652-5p mimic-transfected cell lines was measured by MTS. (E-F) Representative images and the quantitative assessment of colony formation in cells transfected with miR-652-5p mimic. (G-H) Representative images and quantitative measurement of transwell assay in miR-652-5p mimic-transfected cells. (I-J) miR-652-5p induced G1/S phase arrest. Data from triplicate experiments are presented.

Then, we transfected OSCC cells with miR-652-5p inhibitor (S1A Fig). The downregulation of miR-652-5p by the inhibitor induced the malignant phenotypes of TE1 and KYSE510 cells, including cell growth (S1B and 1C Fig), colony formation(S1D and S1E Fig), cell migration and invasion (S1F and S1G Fig). We also found that miR-652-5p downexpression decreased G1 phase cells but increased the number of cells at G2/M phase (S1H and S1I Fig). Therefore, miR-652-5p downregulation could promote the proliferation of OSCC cells.

### miR-652-5p targets PARG and VEGFA to repress proliferation and metastasis

To further investigate the mechanisms by which miR-652-5p mediates the progression of OSCC, we searched for the potential downstream genes of miR-652-5p on bioinformatics databases (i.e. miRDB, miRWalk, and miRTarBase) (Fig 6A). Poly (ADP-ribose) glycohydrolase (PARG) and vascular endothelial growth factor A (VEGFA), two key proteins associated with cell cycling, proliferation, invasion, and metastasis, appeared to be the potential targets of miR-652-5p (Fig 6B). By transfecting EC109 and KYSE150 cells with miR-652-5p mimic, we found that the mRNA and protein expressions of PARG and VEGFA were significantly downregulated compared to the controls (Fig 6C and 6D). On the contrary, the downregulation of miR-652-5p by inhibitor promoted the expressions of PARG and VEGFA at both translational and transcriptional levels (Fig 6E and 6F). To confirm that miR-652-5p directly targeted on PARG and VEGFA, fragments containing the binding sequence of miR-652-5p (or a mutated sequence) in the PARG and VEGFA 3’UTR were cloned into the vectors followed by the co-transfection with miR-652-5p mimic or control miRNA into OCSS cells. The miR-652-5p mimic effectively inhibited the luciferase activities of PARG- or VEGFA-3’UTR (Fig 6D and 6H), whereas control miRNAshowed no effect on them. The inhibition of miR-652-5p on PARG- or VEGFA-3’UTR was sequence-specific as mutant PARG or VEGFA did not decrease the luciferase activities in miR-652-5p mimic-transfected cells. The above results implied that miR-652-5p directly targeted PARG and VEGFA.

**Fig 6:** PARG and VEGFA are the direct targets of miR-652-5p. **(A-B)**PARG and VEGFA were predicted and verified as the targets of miR-652-5p. **(C-D)** The expressions of PARG and VEGFA in EC109 and KYSE150 cells transfected with miR-652-5p mimic were measured by qRT-PCR and western blot. **(E-F)** The mRNA and protein expressions of PARG and VEGFA in EC109 and KYSE150 cells transfected with miR-652-5p inhibitor were measured by qRT-PCR and western blot, respectively. **(G-I)** The luciferase activities in OSCC cells were detected after the co-transfection of miR-652-5p mimic and vectors containing WT or MUT 3’-UTR of PARG and VEGFA. Data from triplicate experiments are presented.

Next, we performed a rescue experiment to ascertain that miR-652-5p targeted on PARG and VEGFA. The endogenous expressions of PARG and VEGFA in EC109 and KYSE150 cells were inhibited by miR-652-5p mimic but recovered by the delivery of PARG- or VEGFA- overexpression constructs (S2A and S2B Fig). The mimic transfection-induced cell migration/invasion was also reversed by the transfection of overexpression constructs (S2C and S2F Fig). Moreover, PARG and VEGFA were silenced in siRNA-transfected cells as shown by significantly attenuated expressions at both mRNA and protein levels (S2G and S2I Fig). The migration/invasion ability of OSCC cells was significantly improved after the silencing of PARG or VEGFA (S2H and S2J Fig). These data indicated that mimic transfection-stimulated cell migration/invasion was reversed by the transfection of either overexpression construct.

### miR-652-5p suppresses tumour progression and metastasis in mice

Furthermore, we assessed the effect of miR-652-5p on OSCC progression in mice. KYSE510 cells were transfected with vectors to knockdown miR-652-5p or control vectors (Fig 7A). The knockdown of miR-652-5p in KYSE510 cells was confirmed by qRT-PCR. KYSE510 cells were then subcutaneously injected in nude mice. Starting on day 7 post-injection, tumour widths and lengths were recorded every five days for 32 days. A significantly increased growth rate was shown in mice inoculated with miR-652-5p-deficient cells compared to the controls(Fig 7B). Then tumours were harvested and their exact sizes and weights were measured. The tumours in miR-652-5p-downregulated group were larger compared to the control animals (Fig 7C and 7D).

**Fig 7:** Knockdown of miR-652-5p promoted tumour progression*in vivo*. **(A)**The level of miR-652-5p in KYSE510 cells stably transfected with lenti-inhibitor and control vector. **(B-D)** KYSE510 cells stably underexpressing miR-652-5p were injected subcutaneously into mice(n = 5 per group). Tumour volume and weight were examined using *in vivo* luciferase imaging on the final day of analysis. **(E-F)** Metastatic nodules were shown in bones, brains, lungs, liver, kidneys and adrenal glands of mice inoculated with miR-652-5p-deficient cells or control cells. **(G-I)** Nude mice were subcutaneously injected with KYSE510 cells and synchronously treated with miR-652-5p agomir or control miRNA (n = 5 per group) by local injection to treat tumour every 7 days. Tumour weight and volume were assessed. **(J)** Immunohistochemistry analysis for Ki67, PARG, and VEGFA in tumour tissues from two groups of animals. **(K)** The expressions of PARG and VEGFA in OSCC tissues samples (n = 103) and matched normal tissues (n = 103) were detected by immunohistochemical staining. Data from triplicate experiments are presented.

Luciferase-labelled cells (1×10^6^) were intravenously injected into the tail veins of mice. All animals were sacrificed six weeks after the injection. The brain, bone, adrenal gland, lung, kidney, and liver metastasis burdens were markedly increased in the group injected with miR-652-5p-deficient cells compared to the control mice (Fig 7E and 7F), suggesting an important role of miR-652-5p in OSCCgrowth and metastasis in mice. To ascertain the inhibitory effect of miR-652-5p on OSCC *in vivo*, we established a mouse OSCC model using KYSE510 cells as above mentioned. Seven days later, miR-652-5p agomir or control agomir was injected into the subcutaneous tumour of mice every five days for thirty-five days. Compared to mice received control agomir, tumour weight and volume of animals treated with miR-652-5p agomir were significantly decreased (Fig 7G–7I). These findings indicated that miR-652-5p overexpression successfully compromised the tumourigenicity of KYSE510 cells in a mouse model.

At last, the proliferative activity of tumour cells was examined by immunohistochemistry staining for Ki-67. Decreased Ki-67 expression was observed in the tumour sections from miR-652-5p agomir-treated group (Fig 7J). MiR-652-5p agomir-treated group also showed attenuated expressions of PARG and VEGFA in the IHC slides as compared to the controls (Fig 7J). Also, the expressions of PARG and VEGFA were significantly upregulated in tumour samples compared to non-tumour tissues (Fig 7K, S3 Table).

## Discussion

Accumulating studies have presented the crucial roles of miRNAs in the progression of multiple human cancers [19–23]. However, the extensive heterogeneity of cancerscomplicates the identification of therapeutic targets and the elimination of all malignant cells [24]. The problem of how to improve the accuracy and efficiency of specific target molecules in cancer treatment remains unsolved[24]. Here, we found that low miR-652-5p expression was an important biomarker that discriminated OSCC tissues from normal tissues. Its correlation with the clinicopathological characteristics suggested that the downregulation of miR-652-5p was associated with OSCC progression. The downregulated miR-652-5p level was also significantly associated with lymph node metastasis and more advanced stages of OSCC. Ourfindings are consistent with recent publications, whichshowed the downregulation of tumour-suppressing miRNAs in OSCC [25,26].

The potential use of endogenous circulating miRNAs in the metastasis, diagnosis, and prognosis of malignancies has been widely reported. Research focusing on serum miRNAs comprises a promising area for the clinical application of miRNAs. Most miRNAs in blood are present in exosomes and are not degraded by proteases [27], suggesting the potential use of exosomal miRNAs to diagnose abnormal physiological conditions or diseases [28,29]. Our data suggested that the serum level of miR-652-5p level might be used to predict the stages of OSCC because of the decreased level of miR-652-5p in patients with higherstage cancer. We further showed that the AUC of miR-652-5p level was 0.919. These results indicated a great potential of miR-652-5p as a non-invasive diagnostic biomarker in OSCC with high specificity and sensitivity. Consistently, the miR-652-5p level in serum exosomes was reduced in OSCC patients compared with healthy controls, indicating that the circulating miR-652-5p accurately reflected the burden of OSCC. Emerging evidence revealed the possible use of miRNAs in the early detection of human malignancies, such as pulmonary cancer [9], breast cancer [10], and stomach cancer[30]. Taylor *et al*. first demonstrated the upregulation of serum exosomal miRNAs in patients with ovarian cancer [31]. Therefore, exosomal miR-652-5p is likely to be a promising non-invasive biomarker and a targetable factor for OSCC diagnosis. Additionally, we showed that the lower expression of miR-652-5p was correlated with poor OS in OSCC patients. Previous studies have reported the upregulation of circulating miRNAs in oesophageal cancer and their potential as new biomarkers for cancer diagnosis [32,33]. Conversely, reduced expressions of miR-138 and miR-145 have been observed in OSCC tissues [34,35]. The current study is the first to demonstrate the prognostic and diagnostic potential of miR-652-5p in OSCC. DNA hypermethylation-mediated inactivation of miRNAsis a key mechanism of tumorigenesis by silencing tumour suppressor genes [36–39]. We hypothesized that the downregulation of miR-652-5p was epigenetically silenced by DNA hypermethylation. The hypermethylation of CpG sites in miR-652-5p was found in OSCC clinical samples. Further analysis verified that 5-aza-CdR-stimulated hypermethylation dramatically augmented miR-652-5p expression in OSCC cells. The above data support the notion that DNA hypermethylation led to reduced miR-652-5p expression during the development of OSCC. This is the first study to present the regulation of DNA methylation on miR-652-5p expression.

Excessive cell proliferation is a fundamental hallmark in cancer progression [40]. It has been demonstrated that miRNAs play crucial roles in tumour cell proliferation [41]. Consistent with these findings, we found that miR-652-5p overexpression suppressed the proliferation, migration/invasion, and colony formation of OSCC cells. The upregulation of miR-652-5p resulted in significant S phage reduction and G0/G1 arrest in OSCC cells. More importantly, miR-652-5p expression in the tissue samples of metastatic OSCC patients was lower in contrast to non-cancerous or non-progressive OSCC tissues. The reduced expression of miR-652-5p stimulated tumour progression in mice, whereas the administration of miR-652-5p agomir successfully suppressed tumour growth *in vivo*, implying that miR-652-5p might a potential therapeutic target for OSCC. Li *et al*. reported the suppressive impact of miR-377 on OSCC initiation and progression and might be used as a non-invasive diagnostic and prognostic biomarker for OSCC patients [42]. Metastasis is responsible for about 90% of cancer mortality [43]. The involvement of different miRNAs in OSCC metastasis has been previously reported [44]. A study showed that the downregulation of miR-370 was associated with the progression of OSCC and promoted tumour cell proliferation by upregulating PIN1 [26]. MiR-382 acted as a tumour suppressor against OSCC development and metastasis, and might be used as a potential drug source OSCC patients [45]. Consistently, our results suggest that miR-652-5p functions as an OSCC suppressor and may be used to develop new treatment methods for OSCC patients.

A single miRNA can target multiple genes to modulate a signalling network. To further explore the tumour-suppressive role of miR-652-5p in OSCC, we searched for its potential targets. The bioinformatics analysis indicated that miR-652-5p bound to the 3′UTR of PARG and VEGFA to inhibit their expressions. PARG is a key enzyme in the degradation of poly (ADP-ribose) and play fundamental roles in maintaining genomic stability and regulating DNA damage repair [46]. PARG is associated with cellular responses to apoptosis and oxidative stress [47]. Moreover, PARG deficiency sensitizes tumour cells to chemotherapy and radiation [48]. The silencing of PARG inhibited the growth of human colon cancer cells [49] and reduced liver metastases in a murine colon carcinoma model [50]. The oncogenic role of PARG has been also reported in Benzo(a)pyrene (BaP)-induced carcinogenesis [51]. VEGFA was originally discovered as a potent regulator of angiogenesis [52]. Later research showed that VEGFA not only that regulates vascular permeability and angiogenesis, but also involved intumour proliferation and metastasis [53]. Several VEGFA-targeting miRNAs were studied, including miR-205 in breast cancer [54] miR-503 in prostate cancer[55] and miR-199a-3p in hepatocellular carcinoma[56].

## Conclusion

Our study suggest that miR-652-5p may inhibit the growth and metastasis of OSCC via targeting PARG and VEGFA. However, there are limitations in this study. Further investigations are needed to determine whether other potential factors are involved in miR-652-5p-mediated OSCC progression. Moreover, exosomes carry a wide range of molecules, including proteins, miRNA, and mRNAs. Studies on the regulatory effects of soluble factors and/or exosomal contents on miR-652-5p in OSCC tumour microenvironment will be of great importance in the future.

## Materials and methods

### Tissue sample collection

A chip array containing OSCC tissues (n = 93) and non-neoplastic oesophageal tissues (n = 93) was obtained from Outdo Biotech (Shanghai, China). Another 100 paired paraffin-embedded OSCC tissues and matched adjacent normal tissues were collected between 2009 to 2013 from North China University of Science and Technology Affiliated People's Hospital. Plasma samples from 110 OSCC patients and 57 healthy subjects were also obtained from this hospital and stored at -80°C. This study was approved by the Ethics Committee of North China University of Science and Technology Affiliated People’s Hospital. All participants gave informed consent. All patient samples were collected after the diagnosis of pathology and with full written consent.

### Cell culture

Human OSCC cells(KYSE30, EC109, TE1, KYSE510, KYSE450, KYSE180, and KYSE150) were obtained from the Typical Culture Cell Bank of Chinese Academy of Sciences (Shanghai, China) and the Cell Culture Centre of Peking Union Medical College (Beijing, China). HEK 293T cells were ordered from ATCC (Manassas, USA). OSCC cells were maintained in RPMI-1640 medium and HEK 293T cells were cultured in DMEM supplemented with 10% foetal bovine serum (FBS, Gibco BRL, Grand Island, USA) in a 5% CO_2_ humidified incubator at 37°C.

### In situ hybridization (ISH)

ISH was performed under RNase-free condition (Roche Molecular Systems, Pleasanton, USA). The probe of miR-652-5p (*5’-TGAATGGCACCCTCTCCTAG-3’*) was tagged with the 3’ and 5’ digoxigenin (Redlandbio, Guangzhou, China). Scrambled control sequence (*5′-GTGTAACACGTCTATACGCCCA-3′*) and U6 snRNA (*5’-CACGAATTTGCGTGTCATCCTT-3’*) were used as negative and positive controls, respectively. Samples were treated with proteinase K (15 μg/ml) for 10 min, washed with PBS, and then sequentially dehydrated by ethanol at increasing concentrations. Then miR-652-5p probe was added into specimens and incubated for one hour at 60°C. After three washes with pre-warmed 5×, 1× and 0.2× SSC, specimens were incubated with the primary anti-DIG antibody for one hour at room temperature and with substrate NBT/BCIP for 15 min in the dark. KTBT was added into the samples to stop further reaction when a blue signal was observed. Samples were classified based on the intensity of cytoplasmic miR-652-5p. High: strong to moderate expression in most cells; low: moderate expression in < 50% of the cells or low expression in most cells; negative: faint or negative expression in most cells.

### Exosome isolation and miRNA extraction from exosomes

Exosomes were isolated from the serum samples of all subjects by differential centrifugation following manufacturer's instructions (RiboBio, Guangzhou, China). In brief, plasma samples were differentially centrifuged at 300×, 1200×, and 10,000× g for three hours. Then the supernatant was filtered and ultracentrifuged at 110,000× g for three hours. Exosomes were harvested from the pellet and resuspended in phosphate-buffered saline (PBS). Exosomal markers CD81and CD63 were detected by monoclonal antibodies (BD Biosciences, Franklin Lakes, USA) using Accuri C6 Flow cytometry (Becton, Dickinson and Company, New Jersey, USA). The sizes of the exosomes were measured by using ZETASIZER Nano series-Nano-ZS (Malvern, England).

### DNA isolation and bisulphite modification

DNA was extracted from OSCC cells, frozen OSCC tissues (n = 18) and paired adjacent normal tissues (n = 18). Purified bisulphite-converted DNAs were tested with human miR-652-5p primers (forward, *5′- aggaagagagTTGGTATTTTGATGAAGAAAGTATTGA-3′*; reverse, *5′-cagtaatacgactcactatagggagaaggctCCTAAAACCAAATTAAACAAAAACT-3′*). The converted DNA was measured using a NanoDrop 2000 spectrophotometer (Thermo, USA). Transformed DNAswere amplified by PCR using the TaKaRa Taq Kit (R001B, TaKaRa, Dalian, China).

### DNA methylation analysis

The sequences of the CpG sites were identified using the UCSC genome browser. The primer set for the methylation analysis was designed by EpiDesigner. An additional T7 promoter tag was added to all reverse primers. A 10-mer tag was added for the forward primer. MiR-652-5p methylation was quantified using the MassARRAY platform (Agena Bioscience Inc.). The DNA methylation level was detected using the matrix-assisted laser desorption/ionization time-of-flight mass spectrometry combined with the base specificity of enzyme reaction. EpiTyper 1.0.5. was used to generate the methylation proportion of each unit. Readings that were not applicable were eliminated from analysis. The level of methylation = methylated cytosines/total cytosines × 100%.

### Epigenetic modulation in cells

OSCC cells were treated with 5-aza-CdR (1.5 mM, Sigma A3656) for ninety-six hours. Trichostatin A (Sigma T8552) at 0.5 mM was added 24 hours before harvest. RNA, DNA, and proteins were isolated and analysed to determine the methylation status of miR-652-5p and the expressions of miR-652-5p and its target genes.

### miRNA transfection

MiRNA mimics(50 nmol/L), agomirs, and inhibitors (100 nmol/L)(RiboBio, Guangzhou, China) were transfected into cells using Lipofectamine 2000 (Invitrogen, Carlsbad, USA). At forty-eight hours post-transfection, cells were harvested for further analyses.

### siRNA transfection

The siRNAs for PARG (*GUUAUCAGUCUGAGCCAGG*) and VEGFA (*GUUAUCAGUCUGAGCCAGG*) were synthesized (RiboBio) and transfected individually into OSCC cells using Lipofectamine RNAiMAX (Invitrogen) at indicated concentrations. To concurrently inhibit the target gene, cells were transfected with a mixture of siRNAs (70 nM in total, 10 nM of each siRNA) or nonspecific control siRNAs (70 nM).

### Plasmid construction

Plasmids (pDonR223-PARG and pDonR223-VEGFA) containing human RB1 and TP53INP1 genes (Axybio Bio-Tech, Changsha, China) were used for the amplification of the coding sequences of PARG and VEGFA. The pEGFP-N1 plasmid, PARG and VEGFA sequences were digested by Hind III and Xho I. Then the fragments were ligated by T4 DNA ligase and transformed into TOP10 competent cells. The positive clones were named as pEGFP-N1-PARG and -VEGFA.

### Quantitative real-time PCR (qRT-PCR)

qRT-PCR was performed to assess the expressions of miR-652-5p, total RNAs, PARG and VEGF for the reverse transcription reactions using a Step One Plus real-time system (AB Applied Biosystems, Carlsbad, USA). The primers were listed in S4 Table. GAPDH and U6 were used as internal controls.

### Luciferase reporter assay

The 3’-UTRs of human PARG and VEGFA were amplified and inserted individually into the pmiR-RB-REPORT (Ribobio) at XhoI and NotI sites. The mutant sequences were inserted into the control vector. OSCC cells were co-transfected with miR-652-5p mimics (or control miR) and PARG- and VEGFA-3′UTR (or PARG- and VEGFA-mut). The luciferase activity was detected forty-eight hours after transfection using a luciferase reporter assay kit (Promega, Madison, USA).

### Cell proliferation assay

Cells (5 × 10^3^ cells/well) were plated and transfected as above mentioned. MTT assay was performed at 0-, 24-, 48-, 72-, and 96-hour. MTT reagent (10 μL) was added to each well. After a 2-hour incubation at 37°C, the optical density was read at 450 nm/570 nm using a microplate reader (BioRad, Hercules, USA).

### Colony formation assay

OSCC cells (1 ×10^3^ cells/well) were cultivated in six-well plates and transfected with miR-652-5p mimic (or control mimic) and miR-652-5p inhibitor (or control inhibitor). Ten days later, cells were fixed with formaldehyde (4%) and stained with Giemsa. Cell colonies in which the total number of cells was >50 were counted.

### Transwell migration/invasion assay

The upper chambers of the Transwell plates (BD Science, Bedford, USA) was covered with Matrigel (BD Science, Bedford, USA) and coagulated overnight. Cells (5× 10^4^ cells/mL) suspended in serum-free RPMI-1640 medium were added to the upper chambers, while the lower chambers were filled with medium (800 μL) containing 10% FBS. After 48 hours, cells in the upper chambers were wiped out with a cotton swab and stained with crystal violet. The migrated cells were counted under 9 randomly-selected fields.

### Flow cytometry

Flow cytometry was performed at 48-hour post-transfection. Cells were fixed in 70% ethanol, stained with propidium iodide (50 μg/mL, 4ABio, China), and analysed using a FACS Calibur flow cytometer (BD Bioscience, USA) and ModFit software (BD Bioscience).

### Western blot

RIPA buffer containing protease and phosphatase inhibitors (Roche) was used to extract total proteins from cells. Cell lysates at equal amounts were separated by SDS-PAGE and then transferred to PVDF membranes (Millipore, USA). After blocking, membranes were incubated with anti-PARG, anti-VEGFA and anti-GAPDH (ab26403, ab1316, ab8245, Abcam, Cambridge, UK) followed by the staining with a goat anti-mouse secondary antibody (1:2000) and a goat anti-rabbit secondary antibody (1:3000). The bands were anlayzed using LAS-4000 Image Reader (Fujifilm) and Multi Gauge V3.2 software.

### Stable cell line generation

Recombinant lentiviral vectors containing the overexpression sequence of miR-652-5p and irrelevant sequence (negative control) were ordered from XIEBHC Biotechnology (Beijing, China). A luciferase and puromycin reporter gene with an EF1α promoter was used to indicate infection efficiency. The miR-652-5p precursor sequence and irrelevant sequence were inserted into the lentiviral vectors, which were then packaged by the co-transfection of HEK 293T cells with pMD2.G and pSPAX2 using LipoFiter reagent. Lentiviral particles were harvested at forty-eight and seventy-two-hour post-transfection and filtered through a 0.45μm cellulose acetate filter (Millipore). After ultracentrifugation, concentrated recombinant lentiviruses were transduced into PSCC cells (MOI ≈5)with polybrene (5 μg/mL) to establish stable cell lines. After 24 hours, the supernatant was replaced by fresh culture medium. The infection efficiency was evaluated using RT-PCR at 96-hour post-infection. Cells were selected with puromycin (2 μg/mL) for fourteen days.

### Tumorigenesis and metastasis *in vivo*

All animal studies were performed following the NIH “Guide for the Care and Use of Laboratory Animals” and the Animal Experimental Guidelines for Biomedical Research Institutes. The potential tumorigenic and metastatic effects of miR-652-5p on OSCC were investigated in the mouse models of subcutaneous and metastasis. In the subcutaneous model, BALB/c nude mice (4-6-week old) were subcutaneously injected with transfected cells (1×10^6^) in the right hip. In the metastasis model, transfected cells (1×10^6^) were injected into the tail vein. After five weeks, tumour colonies in subcutaneous tissues were examined using H&E staining. Bioluminescence images were captured to evaluate the growth and metastasis of tumour cells. Briefly, mice were anaesthetized with isoflurane followed by the intravenous injection of D-luciferin solution (150 mg/kg,PerkinElmer). After 2–5 minutes, the images were acquired with an IVIS Spectrum imaging system (PerkinElmer) and quantified by the Living Image Software (Perkin Elmer/Caliper Life Sciences). The photon flux around the bioluminescence signal was measured(photons/s/cm^2^/steradian).

### Treatment with Agomir

The miR-652-5p agomir and its corresponding control were synthesized by RiboBio. The agomir (10 nmol) and control in 0.1 mL saline were injected to the OSCC cell-forming tumours every five days for six weeks. Tumours were then harvested for immunohistochemistry analysis. The tumour size was monitored by assessing the width (W) and length (L) every five days. The volume was calculated as (L×W^2^)/2. On day 42, animals were sacrificed and the tumours were harvested for RNA and protein extractions.

### Immunohistochemistry examination

Samples were deparaffinised, boiled in citrate buffer (10 mM, pH 6.0), and treated with 3% H_2_O_2_to block endogenous peroxidase. After blocking in serum, slides were incubated with designated antibodies overnight, stained with an anti-rabbit secondary antibody, and visualized using diaminobenzidine (Sigma). IHC images were acquired with a microscope (Olympus) at 200×.The expressions of PARG and VEGFA were scored semi-quantitatively in accordance with the percentage of positively stained cells and the intensity of cytoplasmic/nuclear staining. The percentage of positive cells was: 0 (less than 5%), 1 (6–25%), 2 (26–50%), 3 (51–75%), and 4 (above 75%). The intensity of cytoplasmic/nuclear staining was: 0, negative; 1, buff; 2, yellow; and 3, brown. The optimal cut-off value for this examination system was identified as follows: low expressions: index score < 5; high expressions: index score = 5. Results were independently evaluatedby two investigators.

### Statistical analysis

All cell culture experiments were repeated three times. All data were analysed expressed as means ± SD (SPSS 16.0, SPSS Inc., USA). Statistical significance was evaluated by Student’s t-test, repeated measures ANOVA and χ2 test. The log-rank test was used to analyse the effects of miRNAs and clinical features on the OS. The effect of related factors on the survival time was determined using a Cox regression model. Receiver operating characteristic (ROC) curve was used to evaluate the potential use of serum miR-652-5p as a diagnostic tool for OSCC detection. Cluster 3.0 and Tree View software were used for the stratified cluster analysis of miR-652-5p methylation. Wilcoxon’s test was used to compare the expression of miR-652-5p between OSCC and normal oesophageal tissues. *P*<0.05 was considered statistically significant. ^●^*p* < 0.05, ^●●^*p* < 0.01.

### Ethics approval and consent to participate

This study was reviewed and approved by the Ethics Committee of North China University of Science and Technology Affiliated People’s Hospital.

## Supporting information

S1 Fig Knockdown of miR-652-5p induced cell growth, colony formation and migration in OSCC cells. **(A)** The level of miR-652-5p in TE1 and KYSE510 cell lines after the transfection of miR-652-5p inhibitor. (**B-C)** The growth of miR-652-5p inhibitor-transfected cells was measured by MTS. (**D-E)** Representative images of colony formation and the quantitative assessment in cells transfected with miR-652-5p inhibitor. (**F-G)** Representative images of transwell assay and quantitative measurement in cells transfected with miR-652-5p inhibitor. (**H-I)** miR-602 regulated cell cycle at G1/S phase. Data from triplicate experiments are presented.
(TIF)

S2 Fig RB1 and TP53INP1 were the targets of miR-652-5p. **(A-B)** The mRNA and protein expressions of PARG and VEGFA in EC109 and KYSE150 cells co-transfected with plasmids containing PARG and VEGFA sequences,and miR-652-5p mimic. (**C-F)** Transwell assay of cells co-transfected with miR-652-5p mimic and plasmid containing PARG and VEGFA sequences. (**G)** PARG expression and (**H)** transwell assay in EC109 cells transfected with PARG siRNA. (**I)** VEGFA expression and (**J)** transwell assay in KYSE150 cells transfected with VEGFA siRNA. Data from triplicate experiments are presented.
(TIF)

S1 Table Multivariate cox regression analyses of factors associated with the OS of OSCC. (DOC)

S2 Table The serum miR-652-5p level and clinicopathological parameters of patients with OSCC. (DOC)

S3 Table Correlation between PARG and VEGFA expressions and clinicopathological characteristics of OSCC patients. (DOC)

S4 Table Sequences of primers. (DOC)
